The article "MicroRNA-610 suppresses osteosarcoma oncogenicity via targeting TWIST1 expression" was retracted in 2025. Reasons: manipulated images; plagiarized images; duplicated images; overlap with other authors' work.

# MicroRNA-610 suppresses osteosarcoma oncogenicity via targeting TWIST1 expression

**DOI:** 10.18632/oncotarget.17045

**Published:** 2017-04-11

**Authors:** Chi Jin, Yongjian Feng, Yongjian Ni, Zhonglin Shan

**Affiliations:** ^1^ The Third Department of Orthopaedics, Central Hospital of Cangzhou City, Cangzhou, Hebei, China; ^2^ The Fourth Department of Orthopaedics, Central Hospital of Cangzhou City, Cangzhou, Hebei, China

**Keywords:** osteosarcoma, microRNAs, miR-610, Twist1, cisplatin

## Abstract

Osteosarcoma is the most frequent primary bone tumor affects adolescents and young adults. Recently, microRNAs (miRNAs) are short, non-coding and endogenous RNAs that played as important roles in the initiation and progression of tumors. In this study, we try to explore the biological function and expression of miR-610 in the osteosarcoma. We showed that miR-610 expression was downregulated in the osteosarcoma tissues and cell lines. Elevated expression of miR-610 suppressed the osteosarcoma cell proliferation, cell cycle, invasion and EMT program. Moreover, overexpression of miR-610 increased sensitivity of MG-63 and U2OS cells to cisplatin. Twist1 was identified as a direct target gene of miR-610 in the osteosarcoma cell. Furthermore, we demonstrated that Twist1 was upregulated in the osteosarcoma tissues and cell lines. The expression of Twist1 was negatively associated with the expression of miR-610 expression in the osteosarcoma tissues. Ectopic expression of Twist1 inhibited the sensitivity of miR-610-overexpressing MG-63 cells to cisplatin. We also showed that overexpression of Twist1 increased the proliferation and invasion of miR-610-overexpressing MG-63 cells. These data indicated that ectopic expression of miR-610 suppressed the osteosarcoma cell proliferation, cell cylce, invasion and increased the sensitivity of osteosarcoma cells to cisplatin through targeting the Twist1 expression.

## INTRODUCTION

Osteosarcoma is the most frequent primary bone tumor affects adolescents and young adults, which is prone to early metastasis and frequently occurs in the long bones [1–5]. Despite the recently advancements including adjuvant chemotherapy, radiotherapy and wide tumor excision, the prognosis and 5 years survival rate of these patients remains poor [6–9]. Chemotherapeutic drugs such as cisplatin and doxorubicin are well used in osteosarcoma and 5-year survival rate has been increased from 20% to 70% [10, 11]. However, the molecular mechanisms about acquiring chemoresistance are still unknow [12–14]. It is urgent need to find these molecular mechanisms to explore therapeutic strategies.

MicroRNAs (miRNAs) are a type of short, non-coding and endogenous RNAs that inhibit the protein coding genes expression through partial complementary binding to the 3′ UTR of mRNAs [15–19]. It has been shown that miRNAs mediate several biology functions including cell development, differentiation, apotosis, proliferation, and metabolism [20–24]. Aberrantly expression of miRNAs was found in a variety of human tumors such as gastric cancer, glioblastoma, Ewing's sarcoma, bladder cancer, colon Cancer and also osteosarcoma [16, 25–29]. In addition, mounting evidences demonstrated that miRNAs also act crucial roles in the development of drug resistance in different cancers [30–33].

The article "MicroRNA-610 suppresses osteosarcoma oncogenicity via targeting TWIST1 expression" was retracted in 2025. Reasons: manipulated images; plagiarized images; duplicated images; overlap with other authors' work.

In this study, we try to explore the biological function and expression of miR-610 in the osteosarcoma. We showed that miR-610 expression was downregulated in the osteosarcoma tissues and cell lines. Elevated expression of miR-610 suppressed the osteosarcoma cell proliferation, cell cycle, invasion and EMT program. Moreover, overexpression of miR-610 increased sensitivity of MG-63 and U2OS cells to cisplatin.

## RESULTS

### miR-610 increased the sensitivity of osteosarcoma cells to cisplatin

The miR-610 expression level was downregulated in the osteosarcoma cells (HOS, SAOS-2, MG-63 and U2OS) compared to in the hFOB cells (Figure 1A). qRT-PCR analysis suggested that miR-610 mimic could significantly enhance miR-610 expression both the MG-63 and U2OS cell (Figure 1B and 1C). The response of MG-63 and U2OS cells to cisplatin enhanced after treated with the miR-610 mimic compared to the scramble-transfected cells (Figure 1D and 1E).

**Figure 1:** miR-610 increased the sensitivity of osteosarcoma cells to cisplatin (**A**) The expression of miR-610 in the osteosarcoma cells (HOS, SAOS-2, MG-63 and U2OS) and hFOB cells was determined by qRT-PCR. (**B**) The miR-610 expression in the MG-63 cell after treated with miR-610 mimic. (**C**) MiR-610 mimic could promote the miR-610 expression in the U2OS cell. (**D**) The response of MG-63 cells to cisplatin enhanced after treated with the miR-610 mimic compared to the scramble-transfected cells. (**E**) The response of U2OS cells to cisplatin enhanced after treated with the miR-610 mimic compared to the scramble-transfected cells. *p < 0.05, **p < 0.01 and ***p < 0.001.

### The expression of miR-610 was downregulated in osteosarcoma tissues

We next determined the miR-610 expression level in the osteosarcoma tissues. We showed that miR-610 was downregulated in 21 osteosarcoma cases compare to the adjacent non-tumor tissues (Figure 2A). The miR-610 expression was lower in the osteosarcoma tissues compare with the adjacent non-tumor tissues (Figure 2B).

**Figure 2:** The expression of miR-610 was downregulated in osteosarcoma tissues (**A**) The expression of miR-610 in 30 osteosarcoma cases and adjacent non-tumor tissues was shown. (**B**) The miR-610 expression was lower in the osteosarcoma tissues compare with the adjacent non-tumor tissues.

The article "MicroRNA-610 suppresses osteosarcoma oncogenicity via targeting TWIST1 expression" was retracted in 2025. Reasons: manipulated images; plagiarized images; duplicated images; overlap with other authors' work.

### Overexpression of miR-610 suppressed epithelial-mesenchymal transition (EMT) program

Ectopic expression of miR-610 increased the epithelial marker E-cadherin protein expression and decreased the mesenchymal marker N-cadherin, Vimentin and Snail protein expression (Figure 3A). MiR-610 overexpression promoted the E-cadherin mRNA expression and supressed N-cadherin, Vimentin and Snail mRNA expression (Figure 3B).

**Figure 3:** Overexpression of miR-610 suppressed epithelial-mesenchymal transition (EMT) program (**A**) The protein expression of E-cadherin, N-cadherin, Vimentin and Snail was determined by Western blot. (**B**) The mRNA expression of E-cadherin, N-cadherin, Vimentin and Snail was determined by qRT-PCR.

### Elevated expression of miR-610 suppressed the osteosarcoma cell proliferation

Ectopic expression of miR-610 suppressed the MG-63 and U2OS cell proliferation (Figure 4A and 4B). Moreover, overexpression of miR-610 decreased the ki-67 expression in the MG-63 and U2OS cell (Figure 4C and 4D). In addition, elevated expression of miR-610 supressed the PCNA expression both in the MG-63 and U2OS cell (Figure 4E and 4F).

**Figure 4:** Elevated expression of miR-610 suppressed the osteosarcoma cell proliferation (**A**) Ectopic expression of miR-610 suppressed the MG-63 cell proliferation. (**B**) Overexpression of miR-610 decreased the U2OS cell proliferation. (**C**) The expression of Ki-67 was analyzed by qRT-PCR. (**D**) Ectopic expression of miR-610 suppressed ki-67 expression in the U2OS cell. (**E**) The expression of PCNA was analyzed by qRT-PCR. (**F**) Ectopic expression of miR-610 suppressed PCNA expression in the U2OS cell. *p < 0.05, **p < 0.01 and ***p < 0.001.

### miR-610 overexpression inhibited the osteosarcoma cell cycle and invasion

Ectopic expression of miR-610 suppressed the MG-63 and U2OS cell cycle (Figure 5A and 5B). elevated expression of miR-610 decreased cell invasion both in the MG-63 and U2OS cell (Figure 5C and 5D).

**Figure 5:** miR-610 overexpression inhibited the osteosarcoma cell cycle and invasion (**A**) Ectopic expression of miR-610 suppressed the MG-63 cell cycle. (**B**) MiR-610 overexpression decreased the U2OS cell cycle. (**C**) Elevated expression of miR-610 decreased the MG-63 cell invasion. The relative invasive cells were shown in the right. (**D**) Ectopic expression of miR-610 suppressed the U2OS cell invasion. The relative invasive cells were shown in the right. **p < 0.01 and ***p < 0.001.

The article "MicroRNA-610 suppresses osteosarcoma oncogenicity via targeting TWIST1 expression" was retracted in 2025. Reasons: manipulated images; plagiarized images; duplicated images; overlap with other authors' work.

### Twist1 was a direct target gene of miR-610

To search the molecular mechanism involved in the function of miR-610 in osteosarcoma cell, we used the TargetScan databases to find potential target gene of miR-610. The putative binding site of miR-610 and Twist1 is shown in Figure 6A. Luciferase assay demonstrated that miR-610 overexpression decreased luciferase activity of wild-type (WT) 3′UTR of the Twist1 vector, but not in the mutated-type (Mut) 3′UTR of the Twist1 construct both in the MG-63 and U2OS cell (Figure 6B and 6C). Overexpression of miR-610 suppressed the Twist1 protein expression both in the MG-63 and U2OS cell (Figure 6D and 6E).

**Figure 6:** Twist1 was a direct target gene of miR-610 (**A**) The putative binding site of miR-610 and Twist1 is shown. (**B**) Luciferase report assay demonstrated that miR-610 overexpression suppressed the luciferase activity of wild-type (WT) 3′UTR of the Twist1 vector in the MG-63 cell. (**C**) MiR-610 overexpression suppressed the luciferase activity of wild-type (WT) 3′UTR of the Twist1 vector in the U2OS cell. (**D**) Ectopic expression of miR-610 decreased the Twist1 protein expression in the MG-63 cell. (**E**) The protein expression of Twist1 was measured by western blot. ***p < 0.001.

### Twist1 was upregulated in osteosarcoma tissues

The Twist1 expression level was upregulated in the osteosarcoma cells (HOS, SAOS-2, MG-63 and U2OS) compared to in the hFOB cells (Figure 7A). We furtherly determined the Twist1 expression level in the osteosarcoma tissues. We showed that Twist1 was upregulated in 25 osteosarcoma cases compare to the adjacent non-tumor tissues (Figure 7B). The Twist1 expression was higher in the osteosarcoma tissues compare with the adjacent non-tumor tissues (Figure 7C). The expression of Twist1 was negatively associated with the expression of miR-610 expression in the osteosarcoma tissues (Figure 7D).

**Figure 7:** Twist1 was upregulated in osteosarcoma tissues (**A**) The Twist1 expression in the osteosarcoma cells (HOS, SAOS-2, MG-63 and U2OS) and hFOB was detected by qRT-PCR. (**B**) Twist1 was upregulated in 25 osteosarcoma cases compare to the adjacent non-tumor tissues. (**C**) The Twist1 expression was higher in the osteosarcoma tissues compare with the adjacent non-tumor tissues. (**D**) The expression of Twist1 was negatively associated with the expression of miR-610 expression in the osteosarcoma tissues.

### miR-610 increased the sensitivity of osteosarcoma cells to cisplatin and decreased the osteosarcoma cell proliferation and invasion through downregulating Twist1

The Twist1 mRNA and protein expression was upregulated in the MG-63 cell after tranfected with Twist1 vector (Figure 8A and 8B). The response of MG-63 and U2OS cells to cisplatin enhanced after treated with the Twist1 vector compared to the cotrol-transfected cells (Figure 8C and 8E). Moreover, the responses of miR-610-overexpressing MG-63 and U2OS cells to cisplatin were increased after transfection with the Twist1 vector compared with the control vector (Figure 8D and 8F). Overexpression of Twist1 enhanced MG-63 cell proliferation (Figure 8G) and invasion (Figure 8I). Moreover, ectopic expression of Twist1 promoted the proliferation (Figure 8H) and invasion (Figure 8G) of miR-610-overexpressing MG-63 cells.

The article "MicroRNA-610 suppresses osteosarcoma oncogenicity via targeting TWIST1 expression" was retracted in 2025. Reasons: manipulated images; plagiarized images; duplicated images; overlap with other authors' work.

**Figure 8:** miR-610 increased the sensitivity of osteosarcoma cells to cisplatin and decreased the osteosarcoma cell proliferation and invasion through downregulating Twist1 (**A**) The Twist1 mRNA expression was analyzed by qRT-PCR. (**B**) The Twist1 protein expression was analyzed by western blot. (**C**) The response of MG-63 cells to cisplatin enhanced after treated with the Twist1 vector compared to the cotrol-transfected cells. (**D**) The response of miR-610-overexpressing MG-63 cells to cisplatin was increased after transfection with the Twist1 vector compared with the control vector. (**E**) The response of U2OS cells to cisplatin enhanced after treated with the Twist1 vector compared to the cotrol-transfected cells. (**F**) The response of miR-610-overexpressing U2OS cells to cisplatin were increased after transfection with the Twist1 vector compared with the control vector. (**G**) Overexpression of Twist1 enhanced MG-63 cell proliferation. (**H**) Ectopic expression of Twist1 promoted the proliferation of miR-610-overexpressing MG-63 cells. (**I**) Overexpression of Twist1 enhanced MG-63 cell invasion. (**J**) Ectopic expression of Twist1 promoted the invasion of miR-610-overexpressing MG-63 cells. *p < 0.05, **p < 0.01 and ***p < 0.001.

## DISCUSSION

Osteosarcoma is the most frequent bone tumor occurring in adolescence and childhood, with the high mortality[14, 34, 35]. However, the molecular mechanism about osteosarcoma progression still remains elusive. It is supposed that miRNA deregulated expression is involved in the progression of human tumors[36–39]. In this study, we explored the biological function and expression of miR-610 in the osteosarcoma. We showed that miR-610 expression was downregulated in the osteosarcoma tissues and cell lines. Elevated expression of miR-610 suppressed the osteosarcoma cell proliferation, cell cycle, invasion and EMT program. Moreover, overexpression of miR-610 increased sensitivity of MG-63 and U2OS cells to cisplatin. Twist1 was identified as a direct target gene of miR-610 in the osteosarcoma cell. Furthermore, we demonstrated that Twist1 was upregulated in the osteosarcoma tissues and cell lines. The expression of Twist1 was negatively associated with the expression of miR-610 expression in the osteosarcoma tissues. Ectopic expression of Twist1 inhibited the sensitivity of miR-610-overexpressing MG-63 cells to cisplatin. We also showed that overexpression of Twist1 increased the proliferation and invasion of miR-610-overexpressing MG-63 cells. These data indicated that miR-610 acted as a tumor suppressor role in the osteosarcoma progression and was associated to the sensitivity of osteosarcoma cell to cisplatin.

The article "MicroRNA-610 suppresses osteosarcoma oncogenicity via targeting TWIST1 expression" was retracted in 2025. Reasons: manipulated images; plagiarized images; duplicated images; overlap with other authors' work.

Previous data demonstrated that miR-610 was involved in tumor initiation and progression [40–42]. For example, Wang et al. [40]. suggested that miR-610 suppressed the gastric cancer cell migration and invasion through inhibiting vasodilator-stimulated phosphoprotein (VASP) expression. Zeng et al. [43]. confirmed that miR-610 was decreased in the hepatocellular carcinoma tissues and cell lines. Ectopic expression of miR-610 reduced the hepatocellular carcinoma cell proliferation and tumorigenicity through regulating the protein 1 (TBL1X) and lipoprotein receptor-related protein 6 (LRP6) expression. Mo et al. [42]. showed that the expression level of miR-610 was downregulated in the glioblastoma cell and tissues and overexpression of miR-610 suppressed the glioblastoma cell proliferation through regulating the CCND2 and AKT3 expression. Sun et al. [41]. found that miR-610 expression level was downregulated in the colorectal cancer tissues and overexpression of miR-610 decreased the colorectal cancer cell proliferation, invasion and migration by regulating the hepatoma-derived growth factor (HDGF) expression. Yan et al. [44]. also showed that miR-610 expression was decreased in glioma samples and overexpression of miR-610 suppressed the glioma cell proliferation, invasion and migration by targeting the MDM2 expression. In line with these data, we also demonstrated that miR-610 expression was downregulated in the osteosarcoma tissues and cell lines. Elevated expression of miR-610 suppressed the osteosarcoma cell proliferation, cell cycle, invasion and EMT program.

To study the potential mechanism about miR-610 regulated the proliferation and invasion of osteosarcoma, we used open-target prediction programs (TargetScan databases) to predict the target gene of miR-610, and Twist1 was focused. Twist1 is a conserved basic transcription factor of helix-loop-helix and regulates cell migration, embryonic morphogenesis and differentiation of myoblast, mesodermal and osteoblast [45–48]. Recently, several studies showed that Twist1 played as an oncogene that increased the tumor cell proliferation, migration and invasion, induced the EMT progression, angiogenesis and anti-apoptosis [49–51]. Twist1 has been found to be upregulated in a lot of tumors such as gastric cancer, ovarian cancer, breast cancer, bladder cancer and also osteosarcoma [52–56]. Increasing studies suggested that Twist1 was involved in drug resistance of cancer [55, 57, 58]. In our study, we firstly used the TargetScan databases to show that there is a putative binding site of miR-610 and Twist1. Luciferase assay demonstrated that miR-610 overexpression decreased luciferase activity of WT 3′UTR of the Twist1 vector, but not in the Mut 3′UTR of the Twist1 construct both in the MG-63 and U2OS cell. Overexpression of miR-610 suppressed the Twist1 protein expression both in the MG-63 and U2OS cell. Moreover, we also indicated that Twist1 expression level was upregulated in osteosarcoma tissues and cell lines. The expression of Twist1 was negatively associated with the expression of miR-610 expression in the osteosarcoma tissues. Furthermore, we showed that Twist1 decreased the sensitivity of osteosarcoma cells to cisplatin and ectopic expression of Twist1 promoted the osteosarcoma cell proliferation and invasion. We demonstrated that miR-610 overexpression increased the sensitivity of osteosarcoma cells to cisplatin and decreased the osteosarcoma cell proliferation and invasion through downregulating Twist1 expression.

The article "MicroRNA-610 suppresses osteosarcoma oncogenicity via targeting TWIST1 expression" was retracted in 2025. Reasons: manipulated images; plagiarized images; duplicated images; overlap with other authors' work.

In summary, our study suggested that miR-610 expression level was downregulated in the osteosarcoma samples and cell lines. Ectopic expression of miR-610 suppressed the osteosarcoma cell proliferation, cell cylce, invasion and increased the sensitivity of osteosarcoma cells to cisplatin through targeting the Twist1 expression.

## MATERIALS AND METHODS

### Tissues, cell lines cultured and transfection

Osteosarcoma and the matched adjacent non-tumor tissues were obtained from surgical resection in our hospital. Tissues are immediately frozen in the liquid nitrogen and stored until used. This project was approved with the Institutional Ethics Committee of Central Hospital of Cangzhou City and written informed consent was get from each patient. The Osteosarcoma cell lines (MG63, HOS, U2OS, and Saos-2) and normal human osteoblastic cell line hFOB were cultured in the DMEM (Dulbecco's modified Eagle's medium) suppled with FBS, penicillin and streptomyc. miR-610 mimic and oligonucleotide scramble were obtained from the GenePharm (Shanghai, China) and transfected into the MG-63 cells by using Lipofectamine 2000 (Invitrogen, CA, USA) following to the manufacturer's protocol. These characteristics of patients are described in Supplementary Table 1.

The article "MicroRNA-610 suppresses osteosarcoma oncogenicity via targeting TWIST1 expression" was retracted in 2025. Reasons: manipulated images; plagiarized images; duplicated images; overlap with other authors' work.

### Quantitative RT-PCR

Total RNA was prepared from cells or tissues with TRIzol (Life Technologies, NY). Quantification for miR-610 and TWIST1 was performed by using qRT-PCR following to the manufacturer's information. The expression of U6 was used as the internal control to the expression of miR-610; the expression of GAPDH was used as the internal control to the expression of TWIST. TWIST, forward primer: 5′-ACGAGCTGGACTCCAAGATG-3′ and reverse primer: 5′-CACGCCCTGTTTCTTTGAAT-3′; GAPDH, forward primer: 5′-GACTCATGACCACAGTCCATGC-3′; and reverse primer: 5′-AGAGGCAGGGATGATGTTCTG-3′.

### Cell proliferation and colony formation

Cells were cultured in the 96-well and cell proliferation was determined by MTT assay (Promega, Madison, USA) following to the company's instruction. Cells proliferation was counted after 24 and 48 hours. The absorbance was measured by the microtiter plate reader at 450 nm (Molecular Devices, CA, USA).

### Cell cycle and invasion

For cell cycle analysis, cells were fixed with 70% ethanol, re-suspended in the PBS containing Rnase, Triton X-100 and propidium iodide (Sigma). The cell then was analyzed by FACSArray Flow Cytometer (Becton Dickerson, San Jose, CA, USA). For cell invasion, transwell chambers were used. Cells were cultured on the upper chamber with the non-coated membrane (Millipore) in the serum-free media. The lower chamber with the media containing FBS was used as a chemoattractant. The migration cell on the lower chamber was determined using microscope.

### Luciferase report assay

Cells were cultured in the 48-well plates with about 60% confluence. Cell was transfected with miR-610 mimics or scramble and pGL3-TWIST1-3′UTR and PRL-TK by using Lipofectamine 2000 according to manufacturer's instructions. Renilla and firefly luciferase activitie was determined by using the dual-luciferase reporter (Promega, USA).

### Western blot analysis

Proteins were isolated using a RIPA (radioimmunoprecipitation) lysis buffer. Total protein was separated by 12% SDS-PAGE and then transferred to polyvinylidene fluoride (PVDF) membranes (Millipore, USA). After blocked with the nonfat milk, the membrane was incubated with antibodies against TWIST (1:1000, Santa Cruz, USA), GAPDH (1:5000, Santa Cruz, USA). The membrane was measured by ECL reagent (Applygen, Beijing).

### Statistical analysis

Data are shown as mean ± SD. Comparisons between more than two groups were performed with ANOVA and different between two groups was done using Student's *t*-tests. *P* < 0.05 was considered statistically significant.

## SUPPLEMENTARY TABLE


